# The Impact of Air Quality on Cardiovascular Disease in Shanghai

**DOI:** 10.1155/2022/4421686

**Published:** 2022-01-27

**Authors:** Kai Lu, Jiancheng Kang, Guodong Wang

**Affiliations:** ^1^School of Environmental and Geography Sciences, Shanghai Normal University, Shanghai 200234, China; ^2^School of Tourism, Shanghai Normal University, Shanghai 200234, China

## Abstract

Air pollution is an important factor threatening human health. Inhalation of pollutants can cause damage to the cardiovascular system, leading to increased morbidity and mortality of cardiovascular diseases. This paper selects six pollution factors stipulated by the national air quality standards, collects the air quality index data of Shanghai from 2014 to 2017 and the emergency data of cardiovascular disease in a tertiary hospital in the city during the same period, and conducts relevant analysis to explore different air quality conditions, characteristics, and the relationship between pollutants and cardiovascular disease visits. The results show that the seasonal changes of major air pollutants are related to the incidence of cardiovascular disease.

## 1. Introduction

In recent years, with the rapid development of China's economy and the rapid increase of urbanization, the characteristics of air pollution have gradually changed from traditional coal-burning type to compound type. At present, China's air pollution is still very serious, mainly due to the rapid increase in the total emission of motor vehicle exhaust pollutants in the city, the concentration of total suspended particulates in the atmosphere generally exceeds the standard, the sulfur dioxide pollution remains at a high level, and the nitrogen oxide pollution is increasing. Therefore, strengthening the research on the hazards of atmospheric particulate matter is of great significance to the prevention and control of air pollution.

Data show that, in 2016, the global cardiovascular disease deaths reached 17.647 million [1], among which the number of cardiovascular disease deaths in China was 3.975 million [2]. In 2017, the number of patients with cardiovascular and cerebrovascular diseases in my country reached 290 million, and cardiovascular deaths accounted for No. 1 cause of death among urban and rural residents [3]. The threat of cardiovascular disease has greatly affected the lives and survival of residents, bringing a huge burden to the society and economy, and has become a major public health problem in my country.

The World Health Organization estimated in 2006 that 24% of the global disease burden and 23% of deaths could be attributed to environmental factors [4]. Studies have shown that air pollution can cause damage to human respiratory and circulatory systems, promote arrhythmia, and cause heart failure, ischemic heart disease, cardiac arrest, and other diseases, increasing the incidence and death of cardiovascular diseases rate [5].

The fine particulate matter in air pollutants is also an important indicator for assessing air pollution and disease burden. For example, PM2.5 can rapidly infiltrate the lungs and deposit in the alveolar area and accelerate the damage of blood vessels and heart function by triggering mechanisms such as oxidative stress and inflammation, endangering human health. With long-term or short-term exposure to high-concentrations PM2.5 environment, the risk of cardiovascular disease will continue to increase [6]. Therefore, it is particularly important to understand the relationship between cardiovascular diseases and air pollution, identify the environmental causes of cardiovascular diseases, carry out an environmental risk assessment and early warning of cardiovascular diseases, grasp the trend of major cardiovascular diseases, and formulate cardiovascular disease prevention and control strategy.

## 2. Research Materials

In order to carry out a comparative analysis, this study has collected the following data.

### 2.1. Residents' Outpatient and Emergency Treatment Information

The daily outpatient and emergency number of cardiovascular system diseases from January 2014 to December 2017 in a comprehensive tertiary first-class hospital in the urban area of Shanghai has been collected, and the statistics show that, during the period, the number of outpatients and emergency cardiovascular outpatients in a hospital in Shanghai was 37817 cases; among them, 17,281 were males, accounting for 45.7% of the total number of doctors, and 20536 were females, accounting for 54.3% of the total number of doctors; the male to female ratio was 1 : 1.19.

### 2.2. Air Pollutant Concentration Data

The data of routine observations of air pollutants in urban areas of Shanghai from January 2014 to December 2017 have been collected from the environmental monitoring department.

Observation data include the average AQI, the daily average concentration of PM10, PM2.5, SO_2_, NO_2_, O_3_, and CO, which are the arithmetic averages of data from multiple monitoring points in the urban area.

### 2.3. Data on Social and Economic Development in Shanghai

Relevant data such as Shanghai's GDP information from 2003 to 2018, total industrial waste gas emissions, soot emissions, waste gas sulfur dioxide emissions, the number of days with good ambient air quality and the good rate, energy consumption, the number of deaths from diseases, the number of registered population, the number of permanent residents, the life expectancy of the registered population, and other data have been collected from the Shanghai Bureau of Statistics (Shanghai Statistical Yearbook).

### 2.4. Climate and Environment Characteristics

Shanghai is located on the southeast coast, with a subtropical monsoon oceanic climate with sufficient sunshine and abundant rainfall; the climate is mild and humid; spring is warm, summer is hot, autumn is cool, and winter is cold; spring and autumn are shorter, and winter and summer are longer. Affected by the monsoon, the wind speed in spring is low, mainly easterly; in summer, it is affected by subtropical high pressure, mainly southerly and southeast wind, with higher wind speed; autumn and winter mainly are affected by the Siberian high, with mostly northerly wind at higher speed (10 ms). Throughout the year, the dominant wind direction in Shanghai is the southeast wind, and PM2.5 and PM10 are affected by regional transportation and secondary generation and generally show a distribution pattern of high in the west and low in the east; SO_2_ fully meets the standard, and the concentration is generally low; NO_2_ is generally in the city center. With a decreasing trend to surrounding areas, the concentration in Puxi is generally higher than that in Pudong [6].

### 2.5. Shanghai's Economic Development and Environmental Conditions

Judging from the 2003–2017 Shanghai Economic and Energy-related data from the Shanghai Municipal Bureau of Statistics (see Figure 1), Shanghai's socioeconomic development has been rapid in the 21st century. Between 2003 and 2017, the GDP has increased 4.5 times (increased from 676.238 billion yuan to 3063.299 billion yuan), and the industrial output value has tripled (increased from 1,170.849 billion yuan to 3,609.436 billion yuan). Judging from the data of Shanghai's registered population and permanent population at the end of the year (source: Shanghai Statistical Yearbook), the growth rates were 8.4% and 37%, respectively; with the advancement of technology and the improvement of medical standards, the health of residents has been well protected, life expectancy has been extended, and the average life expectancy of Shanghai's registered population has increased by 3.57 years (increased from 79.80 years old to 83.37 years old), a growth rate of 4.5%, as shown in Table 1.

The above data shows that, with the increase in population and the rapid economic development, energy consumption is also increasing rapidly, as shown in Figure 1. During the 15 years from 2003 to 2017, energy consumption increased by 1.76 times (increased consumption from 67,222,700 tons to 118,589,600 tons), and power resource consumption had more than doubled (increased consumption from 74.597 billion kWh to 152.722 billion kWh). At the same time, the total amount of industrial waste gas emissions also increased significantly, with a growth rate of 77.8%. The overall trend of good air quality and the number of days with good ambient air quality decreased.

In 2012, Shanghai carried out the deployment of the Party Central Committee and the State Council on strict implementation of total pollutant emission control and comprehensively used various methods to continuously increase energy conservation and emission reduction (see Figure 2). With joint efforts, Shanghai smoke and dust emissions from 115,400 tons/year in 2003 dropped to 47,000 tons/year in 2017; the total emission of exhaust gas sulfur dioxide decreased from 435,400 tons/year in 2003 to 18,500 tons/year in 2017; especially beginning from 2013, the total amount of industrial waste gas and sulfur dioxide emissions began to decrease significantly, and the number of days with good ambient air quality and the good rate showed a trend of improvement.

However, comparing the relevant data on pollution emissions and disease deaths in Shanghai from 2003 to 2017, as is shown in Figure 3, we can see that between 2003 and 2017, while the overall trend of respiratory disease mortality has decreased, the growth rates of circulatory system diseases and tumor diseases mortality have reached 43.9% and 23.7%, respectively; the situation is more serious; the reasons and mechanisms for this situation need further study.

The air quality in Shanghai in 2014–2017 was generally good. The number of days with good air quality was 1191 days, with an excellent rate of 81.52%. Especially in 2017, the number of days with good air quality reached 323 days, with an excellent rate of 88.49%; the air quality was seriously polluted. Severe pollution and moderate pollution were mainly concentrated in January, February, November, and December. The number of days of air pollution increased significantly, with 132 days, accounting for 9.03% of the total days. During the same period, the number of cardiovascular visits in hospitals reached 13,553, accounting for a total of 35.84% of the number of cardiovascular visits.

Further comparative analysis of the changes in the air pollution situation and the number of outpatients for cardiovascular diseases in Shanghai from 2014 to 2017 over time (Figure 4) has demonstrated that the pollutant concentration began to rise after autumn, reached the highest peak in winter, and began to decline in spring. When there are many days of air pollution, it is mainly concentrated in winter and early spring. During the period, the concentrations of various pollutants of PM10, PM2.5, SO_2_, NO_2_, CO, and O_3_ all showed periodic changes. PM2.5, NO_2_, and O_3_ did not meet the national average annual second-level standard for environmental air quality, and the pollution problem remained more prominent [7]. Preliminary comparison shows that when the concentration of major pollutants in the air increases, the number of daily outpatient visits for cardiovascular diseases in residents increases accordingly; in cold seasons, the impact of weather pollution on the changes in daily outpatient visits for cardiovascular diseases in residents is bigger than that in warm seasons.

## 3. The Impact of Air Pollution in Shanghai on the Number of Cardiovascular Patients

Air pollution has become an important public health problem on a global scale. It can cause systemic oxidative stress and inflammatory reactions, which can further lead to the hypercoagulable state of human blood, vascular endothelial cell dysfunction, abnormal vasomotor and cardiovascular nerves, regulatory dysfunction, and so on, resulting in toxicity and damage to the cardiovascular system [8].

For Shanghai, a densely populated international metropolis, it is necessary to further explore the relationship between air pollution and cardiovascular disease. To this end, the following subsections discuss the relationship between the content of various air pollutants and the number of visits to cardiovascular diseases.

### 3.1. The Relationship between PM2.5 and the Number of Cardiovascular Patients

PM2.5 refers to particulate matter suspended in the atmosphere with an aerodynamic diameter of less than 25 *μ*m. Its composition may contain toxic components such as polycyclic aromatic hydrocarbons and heavy metals. It has characteristics such as a long atmospheric residence time, which has a significant impact on environmental quality, atmospheric visibility, health, and climate change [9].

A 16-year follow-up study of 500,000 adults conducted abroad by Lee et al. found that, for every 10.5 *μ*g/m^3^ increase in PM2.5, the risk of ischemic cardiomyopathy, arrhythmia, and sudden cardiac death increased by 8%–18% [10]. The “Global Burden of Disease Report 2010” pointed out that China's PM2.5 pollution caused 1.2 million early deaths and 25 million disability-adjusted life-year losses [11]. Research by Dong Ying et al. showed that, between 2014 and 2016, atmospheric PM2.5 pollution caused 6,105 premature deaths and 7,972 hospitalizations for cardiovascular diseases in a certain city [12]. These studies show that there is a definite causal relationship between PM2.5 exposure and cardiovascular disease, and it is a risk factor in the process of cardiovascular events. At present, PM2.5 has become the primary air pollutant in most cities in our country, and it is one of the main bottlenecks to improve ambient air quality, and it has a significant impact on the environment, health, and climate.

Comparing the data of PM2.5 concentration and cardiovascular disease visits in Shanghai from 2014 to 2017, as is shown in Figure 5, we can see that, from March to August, the PM2.5 concentration decreased slightly, and the minimum appeared in August; the growth rate increased significantly, reaching a peak in December. The overall concentration is high in winter and low in summer. The seasons from high to low are winter, spring, autumn, and summer. Compared with the changes in the number of patients for cardiovascular disease during the same period, there is a certain similarity between the two, especially the sharp increase in the number of patients in October and the number of patients starting to decrease after the winter. From March to October, the number of patients and PM2.5 concentration showed a downward trend.

Pollutant particles in the atmosphere mainly affect biological organisms through the respiratory system and gastrointestinal system. PM2.5 and PM10 stimulate the respiratory tract, aggravate asthma, increase the heart rate, reduce lung function, and so on, and tend to affect the respiratory system and cardiovascular system adversely and in severe cases will cause premature death of heart disease patients [13]. Based on the above-mentioned related mechanisms, through active measures such as controlling the level of air pollution and reducing the concentration of PM2.5, the incidence and mortality of cardiovascular diseases can be effectively reduced.

### 3.2. The Impact of PM10 on the Number of Cardiovascular Patients

The particulate matter (PM10) in the atmosphere equal to and less than 10 *μ*m is called inhalable particulate matter; it can absorb a large number of harmful substances such as heavy metal elements and organic pollutants and can enter the gas exchange area in the lung through the human respiratory system, thereby causing the increase of cardiovascular disease morbidity and mortality [14]. A study by Dong and others in Beijing pointed out that, for every 10 *μ*g/m^3^ increase in the concentration of PM10 in the atmosphere, the risk of related cardiovascular diseases increases by 0.63% (95% CI: 0.02%–1.28%) [15]. Studies conducted by Neophytou et al. have pointed out that, for every 10 *μ*g/m^3^ increase in the concentration of PM10 in the air, the death rate of the cardiovascular system increases by 2.43% [16]; it shows that there is a definite relationship between PM10 and cardiovascular diseases.

Checking the relationship between changes in the PM10 concentration in the atmosphere in Shanghai and changes in the number of visits to cardiovascular diseases, as is shown in Figure 6, we can find that, from 2014 to 2017, the PM10 concentration has increased slightly from February, June, and September and reached the peak in December and the minimum appeared in September. The overall appearance is high in winter and low in summer. The seasons from high to low are winter, spring, autumn, and summer. Compared with the changes in the number of patients for cardiovascular diseases, there is a certain similarity between the two, especially when they start in October with the number increasing substantially. From March to October, the number of doctors and PM10 concentration generally showed a downward trend.

### 3.3. The Impact of SO_2_ on the Number of Cardiovascular Patients

SO_2_ is currently one of the most important air pollutants, and the widespread global air pollution caused by it has been highly recognized by all countries. Although China has carried out related treatments against air pollution and has achieved certain results, the current SO_2_ pollution situation in my country is still not optimistic. Cui et al.'s research on Jinan City pointed out that every 10 *μ*g/m^3^ increase in SO_2_ concentration can increase the residents' cardiovascular emergency call events by 0.41% (95% CI: 0.10%–0.72%); the increase in SO_2_ concentration will increase emergency risk of diseases such as blood pressure, coronary heart disease, and stroke [17]. Studies by Sunyer et al. in Europe have also proved that SO_2_ can independently cause cardiovascular disease. The content of SO_2_ in blood and other tissues will increase proportionally with the increase of SO2 concentration in the inhaled air. Long-term exposure to SO_2_ gas can increase the morbidity and mortality of cardiovascular diseases such as arrhythmia, ischemic heart disease, and pulmonary heart disease [18].

Comparing the relationship between the number of visits for cardiovascular diseases and the change of SO_2_ concentration in a Shanghai tertiary hospital, as is shown in Figure 7, we can find that, from the data from 2014 to 2017, the SO_2_ concentration showed a downward trend from January to June, and the minimum appeared in June. The SO_2_ concentration increased from June to December, and the increase began to increase significantly in October and reached its peak in December. As a whole, it shows the characteristics of high in winter and low in summer. The seasons from high to low are winter, spring, autumn, and summer; there is a certain similarity with the changes in the number of patients for cardiovascular disease during the same period. In particular, the number of visits in October increased significantly. From March to October, the number of visits and the concentration of SO_2_ showed a downward trend, and the correlation between the two trends was relatively high.

### 3.4. The Influence of NO_2_ on the Number of Cardiovascular Patients

NO_2_ is a highly insoluble and highly reactive gas, and its emissions are increasing rapidly with the current increase in the number of cars worldwide. The meta-analysis results of Ma Hong et al. showed that, for every 10 *μ*g/m^3^ increase in NO_2_ concentration, the daily mortality risk of residents increased by an average of 1.4% in the short term, and the mortality risk of cardiovascular and cerebrovascular diseases increased by 1.3% [19]. A European study showed that long-term exposure to high concentrations of NO2 would increase the incidence of myocardial infarction disease and has a cumulative dose effect [20]. Research by Cui et al. found that every 10 *μ*g/m^3^ increase in NO_2_ concentration will increase residents' cardiovascular emergency call events by 0.99% (95%CI: 0.27%–1.71%); NO_2_ is associated with heart disease, atrial fibrillation, and hypertension. Coronary heart disease, ischemic heart disease, and other cardiovascular diseases are related [17].

Analyzing the relationship between the number of visits to cardiovascular disease and the change of NO_2_ concentration in a Shanghai tertiary hospital, as is shown in Figure 8, we can find that, from the data from 2014 to 2017, the NO_2_ concentration showed a downward trend in January and April, and NO_2_ from April to August. The concentration continued to decline, and the minimum appeared in August; the increase began to occur significantly in October and reached its peak in December. The overall appearance is characterized by high in winter and low in summer. The seasons from high to low are winter, spring, autumn, and summer; there is a certain similarity with the changes in the number of patients for cardiovascular disease in the same period, especially with the number of patients in October increasing sharply. In autumn and winter, the number of doctors and NO_2_ concentration showed an overall upward trend.

### 3.5. The Impact of CO on the Number of Cardiovascular Patients

CO is the product of incomplete combustion of coal and petroleum containing minerals. It is a colorless, odorless, and nonirritating gas. Under normal circumstances, CO enters the blood through the respiratory system and binds to hemoglobin to participate in the body's metabolism. However, excessive exogenous CO combines with hemoglobin and myoglobin to form carboxyhemoglobin, which inhibits the transport of oxygen, causing hypoxia in the body's cells and even death due to CO poisoning in severe cases [21]. Research in recent years has also found that CO also exists in biological organisms, is widely involved in the physiological and pathophysiological processes of cardiovascular, respiratory, and nervous systems, and exerts biological effects such as anti-inflammatory, antiapoptotic, and antioxidative stress. It has a variety of physiological effects such as relaxation of vascular smooth muscle, antiplatelet aggregation, and regulation of nerves, body fluids, and endocrine involved in the circulatory system; it plays an important physiological role in the occurrence and development of cardiovascular diseases such as hypertension, myocardial injury, arrhythmia, atherosclerosis, and cardiogenic shock [22,23].

Comparing the relationship between the number of visits for cardiovascular diseases in a tertiary hospital in Shanghai and the change of CO concentration, as is shown in Figure 9, we can find that, from the data from 2014 to 2017, the change of CO concentration was relatively mild; from January to June, the CO concentration showed a downward trend. The minimum value appeared in June; after June, the CO concentration began to increase; the increase was obvious in October and reached its peak in December. As a whole, it shows the characteristics of high in winter and low in summer. The seasons from high to low are winter, spring, autumn, and summer in sequence; there is a certain similarity with the changes in the number of patients for cardiovascular diseases. In particular, there has been a substantial increase in the number of patients after October. In general, the number of patients and the overall trend of CO concentration are closely correlated.

### 3.6. The Impact of O_3_ on the Number of Cardiovascular Patients

O_3_ is an active component in atmospheric chemistry. In the tropospheric atmosphere, an appropriate amount of ozone is beneficial to clean the atmosphere. However, due to the increase in the emission of ozone precursors in the troposphere, especially in large cities, the high concentration of ozone produced will cause serious pollution to the atmospheric environment and cause great harm to humans, animals, and the ecological environment [24]. The damage to the cardiovascular system caused by exposure to O_3_ pollutants is also an important factor that air pollution threatens human health. O_3_ has extremely high chemical activity and can participate in many atmospheric photochemical reactions, causing pollution such as acid rain and photochemical smog and directly or indirectly to damage human health. Research by Chen et al. has shown that, for every 10 *μ*g/m^3^ increase in O_3_ mass concentration in the atmosphere, the risk of nonaccidental death in the population increases by 0.79%, and the mortality rate of cardiovascular diseases increases by 1.25% [25]. The study by Atkinson et al. also showed that, for every 10 *μ*g/m^3^ increase in the mass concentration of O_3_ in the air, the death rate of cardiovascular diseases increased by 1.01% [26].

Further analysis of the relationship between the number of visits to cardiovascular disease in a third-class hospital in Shanghai and the change of O_3_ concentration, as is shown in Figure 10, demonstrates that O_3_ pollution is mainly concentrated in spring-autumn. May and September are the peaks of the year, with January and December being the lowest of the year. The characteristic of O_3_ concentration changes is that spring and summer are higher than autumn and winter, and the seasons of concentration from high to low are summer, spring, autumn, and winter. The comparison shows that, in winter and spring, the number of cardiovascular visits decreases with the increase of O_3_ concentration and increases with the decrease of concentration. The low value of O_3_ concentration between the two peaks in July and August is related to the influence of the “Mei Yu” in summer in Shanghai. The rainfall in these two months is relatively large, which reduces solar radiation and inhibits the production of O_3_. Studies abroad have shown that the time distribution of O_3_ concentration is relatively special; the concentration is significantly higher in the high-temperature season than in the low-temperature season, and in terms of spatial distribution characteristics, the closer to the ocean, the higher the concentration, and the closer to the inland, the lower the concentration [27].

### 3.7. AQI and Cardiovascular Disease

AQI (air quality index) describes the degree of air cleanliness or pollution and the impact on human health. In 2012, the Ministry of Environmental Protection included the AQI in the national environmental air quality standard “Ambient Air Quality Standard” (GB3095-2012). The main pollutants involved in air quality evaluation are fine particulate matter, inhalable particulate matter, sulfur dioxide, nitrogen dioxide, ozone, and carbon monoxide.

Figure 11 shows the correlation between AQI and cardiovascular disease. As is shown in Figure 11, from the 2014–2017 AQI data, there are certain seasonal changes; the overall situation is high in winter and spring but low in summer and autumn. The air quality index began to rise in March and August, and the increase occurred significantly in October, reaching a peak in December; there is a certain similarity with the changes in the number of patients for cardiovascular diseases, especially the significant increase in the number of patients in October. After the winter, the number of patients began to decrease. From March to October, the number of patients and the AQI showed a downward trend.

Based on the data of air pollutant concentration and the number of daily outpatients for cardiovascular system diseases in Shanghai from January 2014 to December 2017, correlation and multiple linear regression were used to analyze the difference between the concentration of air pollutants and the number of daily outpatients for cardiovascular diseases. As can be seen from Table 2. PM2.5 has a positive correlation with AQI, PM10, S0_2_, N0_2_, and CO, PM2.5 has a high correlation with AQI and PM10 of 0.958 and 0.918, O3 has a negative correlation with AQI, PM2.5, PM10, S0_2_, N0_2_, and CO. Especially, the negative correlation with CO was as high as −0.837.

At the same time, the correlation between AQI, PM2.5, PM10, S02, N02, CO, O_3_, and the number of cardiovascular outpatient and emergency department visits in a hospital in Shanghai are 0.575, 0.652, 0.597, 0.675, 0.589, 0.568, and −0.508, respectively, which is significant, sexually related; among them, the correlation between AQI, PM2.5, PM10, S02, and female emergency cardiovascular outpatients of a Shanghai hospital is higher than that of male patients, and N02, CO, O_3_, and cardiovascular emergency department in male patients are more relevant than women. A preliminary judgment can be reached that the presence of air pollutants has a certain impact on the incidence of cardiovascular diseases.

Table 3 shows the regression analysis results of the main air pollutants and the number of cardiovascular patients. It can be seen from Table 3 that, through regression analysis, the regression equation of AQI, PM2.5, PM10, S02, N02, CO, and O_3_, and the number of cardiovascular outpatients in a hospital in Shanghai, *Y* is the number of cardiovascular outpatients, and *X* is all indicators for air quality. From the coefficient of determination *R*, it can be judged that the regression equation has a good effect; in the analysis of variance, the significance of Sig is 0.000, less than 0.05, indicating that the regression equation has a strong influence and can well reflect the control relationship between the air quality index and the number of cardiovascular visits.

## 4. Conclusion

The air quality in the Shanghai area is obviously dominated by the number of good days. The seasons with many days of air pollution are mainly concentrated in winter and early spring. The increase in the concentration of the six main pollutants in the air will cause a corresponding increase in the number of daily outpatient visits for cardiovascular diseases in residents; weather pollution has a higher impact on the changes in daily outpatient visits for cardiovascular diseases in the cold season than in the warm season.

The number of cardiovascular visits in a hospital in Shanghai from 2014 to 2017 was significantly correlated with air quality PM2.5, PM10, S02, N02, CO, and O3. Except for the negative correlation of O3, the other indicators of PM2.5, PM10, S0_2_, N0_2_, and CO are positively correlated.. The N02 and CO indicators are positively correlated; they also change with the periodic changes of air quality indicators, showing that the number of cardiovascular visits in winter and spring is significantly higher than that in summer and autumn.

The concentrations of various pollutants of PM10, PM2.5, SO_2_, NO_2_, CO, and O_3_ all show the characteristics of cyclical changes. The concentration of pollutants begins to decrease in spring, and the concentration of pollutants begins to rise after autumn and reaches the highest peak in winter. When there are many days of air pollution, it is mainly concentrated in winter and early spring. The increase in the concentration of major pollutants in the air will cause a corresponding increase in the number of daily outpatient visits for cardiovascular diseases.

It is an indisputable fact that air pollution causes damage to the cardiovascular system, and cardiovascular disease is the leading cause of death for residents worldwide. How to prevent cardiovascular disease and reduce the incidence and death rate of cardiovascular disease has also become a hot topic for related scholars. Only through scientific evidence to enable the general public to understand relevant knowledge as soon as possible, take corresponding protective measures for people at high risk of cardiovascular disease, and at the same time implement actions to increase the control of air pollution, can the morbidity and mortality of cardiovascular disease be reduced, and people's health level and quality of life should be improved.

## Figures and Tables

**Figure 1:** Data on energy consumption in Shanghai from 2003 to 2017 (source: Shanghai Municipal Bureau of Statistics).

**Figure 2:** Data related to air pollution in Shanghai from 2003 to 2017 (source: Shanghai Municipal Bureau of Statistics).

**Figure 3:** Comparison of pollution discharge and disease death data in Shanghai from 2003 to 2017.

**Figure 4:** Data on air pollution and cardiovascular outpatients in Shanghai from 2014 to 2017.

**Figure 5:** Correlation between PM2.5 and the number of patients with cardiovascular disease.

**Figure 6:** Correlation between PM10 and the number of outpatients for cardiovascular diseases.

**Figure 7:** Correlation between SO_2_ and the number of patients in cardiovascular disease.

**Figure 8:** Correlation between NO_2_ and the number of patients in cardiovascular disease.

**Figure 9:** Correlation between CO and the number of patients in cardiovascular disease.

**Figure 10:** Correlation between O_3_ and the number of outpatients for cardiovascular diseases.

**Figure 11:** Correlation between the AQI and the number of patients with cardiovascular disease.

**Table 1:** 2003–2017 Shanghai social, economic, and energy data (source: Shanghai Municipal Bureau of Statistics).

Years	Total industrial output value (100 million yuan)	Shanghai's GDP (100 million yuan)	Energy consumption (10,000 tons of standard coal)	Electricity consumption (100 million kWh)	Population with household registration at the end of the year (10,000 people)	Permanent population (10,000 people)	Life expectancy of registered population (years)
2003	11708.49	6762.38	6722.27	745.97	1341.77	1765.84	79.80
2004	14595.29	8165.38	7303.35	821.44	1352.39	1834.98	80.29
2005	16876.78	9365.54	7974.24	921.97	1360.26	1890.26	80.13
2006	19631.23	10718.04	8604.89	990.15	1368.08	1964.11	80.97
2007	23108.63	12668.89	9374.60	1072.38	1378.86	2063.58	81.08
2008	25968.38	14276.79	9894.52	1138.22	1391.04	2140.65	81.28
2009	24888.08	15287.56	10050.06	1153.38	1400.70	2210.28	81.73
2010	31038.57	17436.85	10671.40	1295.87	1412.32	2302.66	82.13
2011	33834.44	19539.07	10927.62	1339.62	1419.36	2347.46	82.51
2012	33186.41	20558.98	11015.28	1353.45	1426.93	2380.43	82.41
2013	33899.38	22264.06	11345.69	1410.61	1432.34	2415.15	82.47
2014	34071.19	24068.20	11084.63	1369.02	1438.69	2425.68	82.29
2015	33211.57	25659.18	11387.44	1405.56	1442.97	2415.27	82.75
2016	33079.72	28183.51	11712.39	1486.02	1450.00	2419.70	83.18
2017	36094.36	30632.99	11858.96	1526.77	1455.13	2418.33	83.37

**Table 2:** Correlation between major air pollutants and cardiovascular diseases.

		AQI (mean)	PM2.5 (mean)	PM10 (mean)	SO_2_ (mean)	NO_2_ (mean)	CO (mean)	O_3_ (mean)	Number of cardiovascular visits

AQI (mean)	Pearson correlation	1	0.958^*∗∗*^	0.927^*∗∗*^	0.798^*∗∗*^	0.697^*∗∗*^	0.743^*∗∗*^	−0.465^*∗∗*^	0.575^*∗∗*^
	Significance (bilateral)		0.000	0.000	0.000	0.000	0.000	0.001	0.000
	*N*	48	48	48	48	48	48	48	48

PM2.5 (mean)	Significance (bilateral)	0.958^*∗∗*^	1	0.918^*∗∗*^	0.857^*∗∗*^	0.766^*∗∗*^	0.810^*∗∗*^	−0.620^*∗∗*^	0.652^*∗∗*^
	Significance (bilateral)	0.000		0.000	0.000	0.000	0.000	0.000	0.000
	*N*	48	48	48	48	48	48	48	48

PM10 (mean)	Pearson correlation	0.927^*∗∗*^	0.918^*∗∗*^	1	0.854^*∗∗*^	0.747^*∗∗*^	0.713^*∗∗*^	−0.522^*∗∗*^	0.597^*∗∗*^
	Significance (bilateral)	0.000	0.000		0.000	0.000	0.000	0.000	0.000
	*N*	48	48	48	48	48	48	48	48

SO_2_ (mean)	Pearson correlation	0.798^*∗∗*^	0.857^*∗∗*^	0.854^*∗∗*^	1	0.710^*∗∗*^	0.793^*∗∗*^	−0.751^*∗∗*^	0.675^*∗∗*^
	Significance (bilateral)	0.000	0.000	0.000		0.000	0.000	0.000	0.000
	*N*	48	48	48	48	48	48	48	48

NO_2_ (mean)	Pearson correlation	0.697^*∗∗*^	0.766^*∗∗*^	0.747^*∗∗*^	0.710^*∗∗*^	1	0.817^*∗∗*^	−0.735^*∗∗*^	0.589^*∗∗*^
	Significance (bilateral)	0.000	0.000	0.000	0.000		0.000	0.000	0.000
	*N*	48	48	48	48	48	48	48	48

CO (mean)	Pearson correlation	0.743^*∗∗*^	0.810^*∗∗*^	0.713^*∗∗*^	0.793^*∗∗*^	0.817^*∗∗*^	1	−0.837^*∗∗*^	0.568^*∗∗*^
	Significance (bilateral)	0.000	0.000	0.000	0.000	0.000		0.000	0.000
	*N*	48	48	48	48	48	48	48	48

O_3_ (mean)	Pearson correlation	−0.465^*∗∗*^	−0.620^*∗∗*^	−0.522^*∗∗*^	−0.751^*∗∗*^	−0.735^*∗∗*^	−0.837^*∗∗*^	1	−0.508^*∗∗*^
	Significance (bilateral)	0.001	0.000	0.000	0.000	0.000	0.000		0.000
	*N*	48	48	48	48	48	48	48	48

Number of cardiovascular visits	Pearson correlation	0.575^*∗∗*^	0.652^*∗∗*^	0.597^*∗∗*^	0.675^*∗∗*^	0.589^*∗∗*^	0.568^*∗∗*^	−0.508^*∗∗*^	1
	Significance (bilateral)	0.000	0.000	0.000	0.000	0.000	0.000	0.000	
	*N*	48	48	48	48	48	48	48	48

^*∗∗*^Significant correlation at the 0.01 level (bilateral). ^*∗*^Significant correlation at the 0.05 level (bilateral).

**Table 3:** Regression analysis of major air pollutants and cardiovascular visits.

	AQI (mean)	PM2.5 (mean)	PM10 (mean)	SO_2_ (mean)	NO_2_ (mean)	CO (mean)	O_3_ (mean)
Sig	0.0000	0.0000	0.0000	0.0000	0.0000	0.0000	0.0000
*R* ^2^	0.575	0.625	0.597	0.675	0.589	0.568	0.508
And the number of cardiovascular visits (*Y*)	*Y* = 5.466^*∗*^*X* + 382.986	*Y* = 6.216^*∗*^*X* + 497.309	*Y* = 4.746^*∗*^*X* + 497.505	*Y* = 16.83^*∗*^*X* + 547.113	*Y* = 6.911^*∗*^*X* + 489.978	*Y* = 583.663^*∗*^*X* + 320.097	*Y* = −3.456^*∗*^*X* + 1034.544

## Data Availability

The datasets used and/or analyzed during the current study are available from the corresponding author upon reasonable request.
